The article "Glutathione peroxidase 4 plays an important role in oxidative homeostasis and wound repair in corneal epithelial cells" was published in 2016. Journal: FEBS Open Bio.

# Glutathione peroxidase 4 plays an important role in oxidative homeostasis and wound repair in corneal epithelial cells

**DOI:** 10.1002/2211-5463.12141

**Published:** 2016-10-24

**Authors:** Osamu Sakai, Takatoshi Uchida, Hirotaka Imai, Takashi Ueta

**Affiliations:** ^1^ Department of OphthalmologyGraduate School of Medicine and Faculty of MedicineThe University of TokyoJapan; ^2^ Senju LaboratorySenju Pharmaceutical Co. Ltd.KobeJapan; ^3^ School of Pharmaceutical SciencesKitasato UniversityTokyoJapan

**Keywords:** corneal epithelial cell, GPx4, oxidative stress, wound healing

## Abstract

Oxidative stress is involved in the pathologies of corneal epithelial cells. However, the importance of specific antioxidant enzymes in corneal epithelial cells is not fully understood. The purpose of this study is to elucidate the role of glutathione peroxidase 4 (GPx4) in corneal epithelial cells. For *in vitro* experiments, an immortalized human corneal epithelial cell line was used. Cytotoxicity measured through LDH activity, lipid peroxidation immunostained for 4‐hydroxynonenal, cell viability, and cell death were compared between cells transfected with either GPx4 siRNA or scrambled control siRNA. In addition, the rescue effects of α‐tocopherol and ferrostatin‐1, a ferroptosis inhibitor, were examined in the cells with deficient GPx4 expression. For *in vivo* experiments, we applied n‐heptanol on the cornea of GPx4^+/+^ and GPx4^+/−^ mice to create corneal epithelial wound. The epithelial defect area size was measured up to 48 h after epithelial wound creation. Knockdown of GPx4 strongly induced cytotoxicity and cell death in human corneal epithelial cells. Cell death induced by GPx4 knockdown was characterized by positive staining for both annexin V and propidium iodide, nuclear translocation of AIF, and without activation of caspase 3, and was rescued by α‐tocopherol and ferrostatin‐1. The delayed wound healing of GPx4 siRNA‐transfected cells were ameliorated by α‐tocopherol *in vitro*. In addition, loss of one GPx4 allele was sufficient to significantly delay the healing of experimental corneal epithelial wounds *in vivo*. Our results suggest that the antioxidant enzyme GPx4 plays an important role in oxidative homeostasis, cell survival, and wound healing in corneal epithelial cells.

**Abbreviations**
4‐HNE: 4‐hydroxynonenal
AIF: apoptosis‐inducing factor
DMEM: Dulbecco's modified Eagle medium
GPx: glutathione peroxidase
HCEC: human corneal epithelial cell line
LDH: lactate dehydrogenase
PI: propidium iodide
PVDF: polyvinylidene fluoride
SOD: superoxide dismutase

The cornea is constantly exposed to environmental insults, and oxidative stress from these insults is considered to be implicated in corneal diseases 1, 2, 3.

Redox homeostasis is maintained by various antioxidant enzymes including catalase, superoxide dismutase (SOD), and glutathione peroxidase (GPx) 4, 5, 6. Downregulation of the activities or expressions of antioxidant enzymes has been observed in some pathologies 7, 8. Abnormal accumulation of byproducts produced because of oxidative stress has been identified in corneal tissue and in tear fluid of the patients with corneal diseases, such as dry eye, conjunctivochalasis, and atopic keratoconjunctivitis 1, 2, 3, as well as in animal models for pathologies involving corneal epithelium 9, 10, 11. However, despite the importance of the defense mechanism against oxidative stress, which has been widely accepted, the importance of specific antioxidant enzymes in corneal epithelial cells is not fully understood.

GPx4 is one of the eight GPx isozymes found in mammals 6. It is ubiquitously expressed 12 and has a unique substrate specificity that directly reduces peroxidized lipids in cell membrane 13. Lipid peroxidation is implicated in a variety of pathophysiological processes 3, 14, 15, and byproducts of lipid peroxidation, such as 4‐hydroxynonenal (4‐HNE), are known to induce cell damage, including growth inhibition and cell death 16, 17. Conventional GPx4 knockout mice die at embryonic day 8 18. Loss of GPx4 results in lipid peroxidation leading to cell death 19, 20, whereas the overexpression of GPx4 confers protection against oxidative stress‐mediated injury 21, 22.

In this study, we elucidated the importance of GPx4 in corneal epithelial cells *in vitro* and *in vivo*.

## Materials and methods

### Cell culture and transfection of siRNA

Human corneal epithelial cell line (HCEC, SV40‐T Ag‐immortalized human corneal epithelial cell line) that was established by Araki‐Sasaki *et al*. 23 was cultured in Dulbecco's modified Eagle medium (DMEM)/F12 medium with 10% heat‐inactivated FBS (Invitrogen, Carlsbad, CA, USA) and 100 U penicillin plus 100 μg·mL^−1^ streptomycin under 5% CO_2_ at 37 °C. Other selenium source like Na‐selenite was not used in our culture condition.

Cells were transfected with 25 nm siRNA for catalase, GPx1, GPx4, SOD1, SOD2 (Ambion Silencer predesigned siRNA, catalase ID: s2445, GPx1 ID: s804, GPx4 ID: s6112, SOD1 ID: s451, SOD2 ID: s13268), or scramble control siRNA using lipofectamine RNAiMAX (Invitrogen) following the manufacturer's instruction. Morphology of transfected cells was assessed with an inverted phase‐contrast microscope. In some experiments, α‐tocopherol (10 μm) and ferrostatin‐1 (10 μm) was added after 24 h of GPx4 siRNA transfections.

### Real‐time RT‐PCR

Two days after transfection with siRNA, total RNA of the cells was isolated using Isogen (Nippon Gene, Tokyo, Japan) according to the manufacturer's instructions. For the *in vivo* studies, total RNA was isolated from microsurgically dissected mouse cornea in the same manner. Subsequently, RNA was reverse‐transcribed into cDNA by ReverTra Ace^®^ qPCR RT Master Mix with gDNA Remover (Toyobo, Osaka, Japan). Quantitative real‐time PCR was carried out with thermal cycler dice (Takara, Shiga, Japan) using Platinum SYBR Green qPCR SuperMix‐UDG (Invitrogen). The levels of GAPDH were used as the inner control. The sequences of the primers used in the real‐time RT‐PCR were as follows: human GAPDH (Fwd, 5‐TTGATTTTGGAGGGATCTCG‐3 and Rev, 5‐AACTTTGGCATTGTGGAAGG‐3), human catalase (Fwd, 5‐GCCTGGGACCCAATTATCTT‐3, Rev, 5‐GAATCTCCGCACTTCTCCAG‐3), human GPx1 (Fwd, 5‐CTCTTCGAGAAGTGCGAGGT‐3, Rev, 5‐TCGATGTCAATGGTCTGGAA‐3), human GPx4 (Fwd, 5‐GCACATGGTTAACCTGGACA‐3, Rev, 5‐CTGCTTCCCGAACTGGTTAC‐3), human SOD1(Fwd, 5‐TGGCCGATGTGTCTATTGAA‐3, Rev, 5‐GGGCCTCAGACTACATCCAA‐3), human SOD2 (Fwd, 5‐TTGGCCAAGGGAGATGTTAC‐3, Rev, 5‐AGTCACGTTTGATGGCTTCC‐3), mouse GAPDH (Fwd, 5‐CACATTGGGGGTAGGAACAC‐3 and Rev, 5‐AACTTTGGCATTGTGGAAGG‐3), and mouse GPx4 (Fwd, 5‐CGCGATGATTGGCGCT‐3 and Rev, 5‐CACACGAAACCCTGTACTTATCC‐3).

### Immunoblotting

For *in vitro* experiments, cells after 2 days of transfection with siRNA were used. For *in vivo* experiments, the dissected mouse corneas were used. Proteins were extracted from the cells and mouse corneas using LIPA buffer. As previously described 24, SDS/PAGE of the proteins was performed on Mini‐PROTEAN TGX Any kD gel (Bio‐Rad Laboratories, Hercules, CA, USA) with tris‐glycine‐SDS running buffer (Bio‐Rad Laboratories). Immunoblot analysis was performed by electrotransferring proteins from the gels onto polyvinylidene fluoride (PVDF) membranes (Millipore, Billerica, MA, USA) at 100 V for 60 min at ice‐cold temperature using tris‐glycine buffer. The membranes were probed with antibodies to GAPDH (Santa Cruz Biotechnology, Santa Cruz, CA, USA), catalase (Santa Cruz Biotechnology), GPx1 (Cell Signaling Technology, Danvers, MA, USA), GPx4 (Cayman, Ann Arbor, MI, USA), SOD1 (Santa Cruz Biotechnology), or SOD2 (GeneTex, Irvine, CA, USA). Binding of secondary antibodies, conjugated to alkaline phosphatase or to horseradish peroxidase, was visualized with 5‑bromo‐4‑chloroindol‐2‑yl phosphate/Nitro Blue tetrazolium substrate (Bio‐Rad Laboratories) or chemiluminescent substrate (Pierce, Rockford, IL, USA).

### Caspase activity

Activation of caspase was examined by immunoblotting for caspase 3. Three days after transfection with siRNA, immunoblotting was conducted using antibodies to caspase 3 (Cell Signaling Technology) and GAPDH (Santa Cruz Biotechnology) as described above. Cells treated with 1.0 μm staurosporine were also used as a positive control for caspase activity.

### Cytotoxicity assay

Membrane breakage and cell death were quantitated using release of lactate dehydrogenase (LDH) into the culture medium 25. Three days after transfection with siRNA, cytotoxicity by the knockdown of SOD1, SOD2 catalase, GPx1, or GPx4 was evaluated using LDH cytotoxicity detection kit (Takara). LDH activity was measured in the extracellular medium and in the cell lysate according to the manufacturer's instructions, and then extracellular LDH activity was calculated as percentage of the total LDH activity.

### Evaluation of lipid peroxidation

4‐hydroxynonenal is known as a useful biomarker for lipid peroxidation 16, 17, 26 and the assay was performed as described previously 24. After 3 days of transfection with siRNA, cells were fixed with 4% paraformaldehyde for 15 min, washed three times with PBS, and permeabilized with 0.1% of Triton X‐100 solution containing 5% goat serum in PBS. Permeabilized cells were washed three times with PBS containing 5% goat serum, incubated with anti‐4‐HNE antibodies (JaICA, Shizuoka, Japan) for 1 day at 4 °C. Then, cells were washed again three times with PBS. Alexa 488‐conjugated anti‐mouse IgG secondary antibodies (Invitrogen) were applied, the sample left at room temperature for 1 h, and excess antibodies were removed by washing cells three times with PBS. Fluorescent images were observed with a fluorescence microscope (Keyence, Osaka, Japan). The fluorescence intensities of the dots stained with 4‐HNE were quantitated using image j software (NIH, Bethesda, MD, USA).

### Determination of reactive oxygen species

Production of reactive oxygen species (ROS) was determined using an oxidation‐sensitive fluorescent probe, 2′7′‐dichlorofluorescin diacetate (DCFH‐DA). After 4 days of transfection with GPx4 or control siRNA, cells were incubated with 100 μm DCFH‐DA (Invitrogen) for 30 min, and rinsed with viability medium. Then, the fluorescence was analyzed at 485/535 nm excitation/emission.

### Annexin V and propidium iodide staining

Annexin V/Propidium iodide (PI) staining was performed using the FITC Annexin V Apoptosis Detection Kit (BD Bioscience, San Jose, CA, USA). Three days after transfection with siRNA, cells were stained by FITC‐conjugated Annexin and PI for 15 min at room temperature, and washed with PBS. Images were obtained with a fluorescence microscope (Keyence).

### AIF translocation

Apoptosis inducing factor (AIF) is an effector protein for regulated necrosis, and has been shown to translocate from mitochondria to nucleus when cell death is induced 27. Localization of AIF was evaluated by immunostaining using anti‐AIF antibodies (Santa Cruz Biotechnology) after 3 days of transfection with siRNA. Nucleus was stained with 4′,6‐diamidino‐2‐phenylindole. Fluorescent images were obtained with a fluorescence microscope (Keyence).

### Cell viability assay

Cellular viability was assessed using WST‐8 assay (Dojindo, Kumamoto, Japan) at 0, 1, 3, and 5 days after siRNA transfection, following the manufacturer's instructions.

### *In vitro* wound closure assay

*In vitro* wound closure assay was performed based on the previous literature 11, 28. HCEC cells were seeded onto a 24‐well cell culture plate, in which a 7‐mm‐diameter circular seal was affixed to the bottom of each well, and cultured for 24 h. Next, the cells were transfected with siRNA. Two days after transfection, affixed seals were removed from the bottom of each well to generate cell‐free areas of the same size. The cells were cultured for an additional 48 h. Then, the plates were washed two times using PBS, and the cells were fixed with 10% formalin neutral buffer solution. The fixed cells were washed three times using PBS, and stained with 0.05% toluidine blue solution. The bottom of each of the stained experimental wells was photographed, and the remaining wound area size was measured using image j software.

### Corneal epithelial wound healing in mice

We used GPx4^+/+^ and GPx4^+/−^ mice with C57BL/6 background 29. Animals were maintained in ordinary animal cages under constant 12‐h light/dark cycles. Food and water were available *ad libitum*. All animal experiments were performed in accordance with the Association for Research in Vision and Ophthalmology (ARVO) Statement for the Use of Animals in Ophthalmic and Vision Research and the NIH Guiding Principles in the Care and Use of Animals (DHEW Publication, NIH 80‐23), and were approved by the Institutional Animal Research Committee of the University of Tokyo.

Mice were anesthetized by intramuscular injection of a mixture of ketamine and xylazine. Paper filters (2‐mm diameter) soaked in n‐heptanol were attached to the center of each corneal surface for 1 min to remove corneal epithelia, and then the treated eyes were washed with saline. The epithelial defect was stained with 1% fluorescein solution and photographed at 0, 6, 12, 18, 24, 30, 36, 42, and 48 h after epithelial debridement. The area of the epithelial defect was measured on photographs using image j software.

### Statistical analysis

Data were presented as mean ± standard error mean (SEM). Statistical analysis was performed with 2‐tail Student's *t*‐test or one‐way analysis of variance (ANOVA) followed by Tukey's test. *P* < 0.05 was considered statistically significant.

## Results

### Knockdown of antioxidant enzymes

Human corneal epithelial cells were transfected with siRNA to specifically knockdown the expressions of catalase, GPx1, GPx4, SOD1, or SOD2. Two days after transfection, mRNA (Fig. 1A) and protein (Fig. 1B) levels were measured through real‐time RT‐PCR and immunoblotting. The mRNA levels of all the antioxidant enzymes were downregulated by >80%. In addition, a significant downregulation in the protein levels of each antioxidant enzyme was also confirmed.

**Figure 1:** Knockdown of different antioxidant enzymes using siRNA in corneal epithelial cells. (A) Knockdown efficiency evaluated by mRNA levels (*n* = 3–4). (B) Knockdown efficiency evaluated by protein levels using immunoblot analysis. Reproducibility was confirmed in triplicate. (C) Phase contrast morphology of corneal epithelial cells transfected with siRNA of scramble control, catalase, GPx1, GPx4, SOD1, or SOD2 at day 3 after transfection. Scale bar, 50 μm. (D) LDH release from corneal epithelial cells 3 days after transfection with siRNA for scramble control, catalase, GPx1, GPx4, SOD1, or SOD2 (*n* = 4). **P < 0.01 using Tukey's test. (E) Knockdown of GPx4 enhanced LDH release induced by H_2_O_2_ (*n* = 4). **P < 0.01 using Tukey's test.

We examined the morphological characteristics of corneal epithelial cells treated with each targeted siRNA 3 days after transfection (Fig. 1C). Cells transfected with control siRNA showed to be compact, uniform, and cobblestone pavement in shape. The shape of the cells transfected with catalase, GPx1, SOD1, or SOD2 resembled that of cells transfected with control siRNA. Conversely, cells transfected with GPx4 siRNA exhibited signs of cell damage including spheroid structures.

Lactate dehydrogenase activity was evaluated as an indicator of cytotoxicity. Knockdown of catalase, GPx1, and SOD2 did not influence LDH activity (Fig. 1D). Knockdown of GPx4 and SOD1 induced a significant increase in the LDH activity. However, the LDH activity of GPx4 knockdown was significantly higher than that of SOD1 knockdown.

To further clarify the protective effect of GPx4 under oxidative stress conditions, we investigated the effect of GPx4 knockdown on cytotoxicity enhanced by hydrogen peroxide (Fig. 1E). LDH activity of the cells transfected with control siRNA was not influenced by the addition 100 μm hydrogen peroxide. Conversely, LDH activity of the cells transfected with GPx4 siRNA significantly increased after treatment with 100 μm hydrogen peroxide. Knockdown of GPx4 enhanced cytotoxicity under mild oxidative stress, suggesting an important role for GPx4 against oxidative stress.

### α‐tocopherol rescued cytotoxic effects of GPx4 knockdown

α‐tocopherol has been reported to confer protection against cytotoxicity and cell death induced by GPx4 deficiency 20, which we subsequently tested in corneal epithelial cells *in vitro*. Our results show that α‐tocopherol significantly prevented LDH release from cells transfected with GPx4 siRNA (Fig. 2A). Next, we evaluated lipid hydroperoxide generation using immunostaining for 4‐HNE and total intracellular ROS using DCFH‐DA. Results show that both 4‐HNE and total ROS were significantly elevated in cells transfected with GPx4 siRNA, which was rescued by treatment with α‐tocopherol (Fig. 2B–D). Figure 3 shows the cell death induced by GPx4 knockdown. Annexin V and PI staining indicated that most of the dead cells were annexin V positive with PI staining after 3 days of GPx4 silencing while the number of cells with either Annexin V or PI staining only was relatively small. In addition, the cell death was rescued by α‐tocopherol treatment (Fig. 3A).

**Figure 2:** α‐tocopherol rescues cytotoxic effects of GPx4 knockdown in corneal epithelial cells. (A) α‐tocopherol prevented the LDH release induced by GPx4 knockdown (*n* = 4). **P < 0.01 using Tukey's test. (B) Accumulation of 4‐HNE was evaluated by immunofluorescence. Scale bar, 50 μm. (C) Fluorescence intensities for 4‐HNE were quantitated using image j (*n* = 8–9). **P < 0.01 using Tukey's test. (D) Total intracellular ROS was quantitated using DCFH‐DA (*n* = 4). **P < 0.01 and *P < 0.05 using Tukey's test.

**Figure 3:** Cell death caused by GPx4 knockdown in corneal epithelial cells. (A) Representative image of annexin V and PI staining. Majority of the staining was annexin V positive with or without PI staining. Scale bar, 50 μm. (B, C) Nuclear translocation of AIF (green) induced by GPx4 knockdown was evaluated in the total number of cells. 4′,6‐diamidino‐2‐phenylindole was used for nuclear staining (*n* = 6–10). **P < 0.01 using Tukey's test. Scale bar, 50 μm. (D) Caspase‐3 and cleaved caspase‐3 (active form) were immunoblotted for cells transfected with siRNA for scramble control or GPx4. Staurosporin (1 μm) served as a positive control. Reproducibility was confirmed in triplicate. (E) Effect of ferrostatin‐1 (10 μm) to rescue the decreased cell viability induced by GPx4 knockdown. **P < 0.01 using Tukey's test. (F) Effect of ferrostatin‐1 (10 μm) to rescue the increased LDH activity induced by GPx4 knockdown. **P < 0.01 using Tukey's test.

Next, we investigated possible mechanisms for the cell death by GPx4. The percentage of cells with AIF translocation to the nucleus increased in cells transfected with GPx4 siRNA (Fig. 3B,C). Furthermore, α‐tocopherol prevented the AIF translocation induced by GPx4 knockdown (Fig. 3B,C). In contrast, cleaved caspase‐3, implicated in caspase‐dependent apoptosis, was not detected in cells transfected with control siRNA or GPx4 siRNA (Fig. 3D), while staurosporine treatment (positive control) led to the activation of caspase 3. We further examined the implication of ferroptotic mechanism using ferrostatin‐1, an inhibitor of ferroptosis. Ferrostatin‐1 partially ameliorated the decrease in cell viability (Fig. 3E) and the increase in LDH activity (Fig. 3F) caused by GPx4 knockdown.

### Effects of GPx4 knockdown on cell viability

We examined the effects of GPx4 knockdown on corneal epithelial cell growth. First, we evaluated cell viability using WST‐8 assay. There was no significant difference in cell viability between cells transfected with GPx4 and control siRNA up to 1 day after transfection (Fig. 4A). However, at 3 and 5 days after transfection, the viability of GPx4 siRNA‐transfected cells was significantly lower than that of control siRNA‐transfected cells (Fig. 4A), suggesting that GPx4 is essential for growth of corneal epithelial cells.

**Figure 4:** Wound healing model of corneal epithelial cells *in vitro*. (A) Viability was evaluated by WST‐8 assay at day 0, 1, 3, 5, and 7 after transfection (*n* = 5). **P < 0.01 by Student's *t*‐test. (B, C) Cell viability and migration was evaluated in wound healing model *in vitro*. Remaining wound area (% of each initial area) at 48 h after wound creation was compared (*n* = 4). *P < 0.05 and **P < 0.01 using Tukey's test.

Next, we examined the effects of GPx4 knockdown on the wound closure system of corneal epithelial cells *in vitro*. Two days after wound creation, a significant delay in the wound closure was observed in the cells treated with GPx4 siRNA, and α‐tocopherol ameliorated the delay caused by GPx4 knockdown (Fig. 4B,C).

### Corneal epithelial wound healing in GPx4^+/+^ and GPx4^+/−^ mice

We confirmed the decreased expression of GPx4 in both the mRNA and protein level in the cornea of GPx4^+/−^ mice compared to that of GPx4^+/+^ mice (Fig. 5A,B). In line with the decreased GPx4 expression, lipid peroxidation levels in the cornea of GPx4^+/−^ mice were significantly higher than those in the cornea of GPx4^+/+^ mice (Fig. 5C,D). Then, we examined corneal epithelial wound healing in GPx4^+/−^ mice and GPx4^+/+^ mice after topical exposure to n‐heptanol. At 18, 24, 30, and 36 h after n‐heptanol treatment, the remaining epithelial defect area in GPx4^+/−^ mice was larger than that in GPx4^+/+^ mice (Fig. 5E,F). The epithelial defect was resurfaced in all the GPx4^+/+^ mice by 36 h after exposure to n‐heptanol, whereas even at 42 h the defect was not completely resurfaced in GPx4^+/−^ mice.

**Figure 5:** Corneal epithelial wound healing in GPx4^+/−^ and GPx4^+/+^ mice. (A) GPx4 mRNA levels in the cornea of GPx4^+/−^ and GPx4^+/+^ mice (*n* = 5–6). **P < 0.01 by Student's *t*‐test. (B) GPx4 protein levels were determined using western blot. Reproducibility was confirmed in triplicate. (C) Accumulation of 4‐HNE was evaluated by immunofluorescence. Scale bar, 100 μm. (D) Fluorescence intensities for 4‐HNE were quantitated using image j (*n* = 3). *P < 0.05 by Student's *t*‐test. (E) Representative photographs of corneal epithelial wound healing in GPx4^+/−^ and GPx4^+/+^ mice. Green areas represented fluorescein‐stained wounded areas (F) The remaining area size of the wounds (% of each initial wound area) was compared between GPx4^+/−^ and GPx4^+/+^ mice (*n* = 10–12). **P < 0.01 and *P < 0.05 using Student's *t*‐test.

## Discussion

The major contribution of this study is that we show that GPx4 is by itself an important antioxidant enzyme for maintaining redox homeostasis and wound healing in corneal epithelial cells. Decreased expression of GPx4 led to cytotoxicity by oxidative stress, caspase‐independent cell death with nuclear translocation of AIF, and decreased viability and wound healing in corneal epithelial cells. We confirmed that α‐tocopherol could potentially compensate for the lack of GPx4 in corneal epithelial cells.

Oxidative stress and antioxidant system have been intensively discussed in the cornea pathologies 11, 30, 31. However, the importance of a specific antioxidant enzyme has not been fully understood. Degeneration and dysfunction of lacrimal glands leading to age‐related dry eye signs has only been reported in mice deficient of SOD1 9. In the present study, we silenced the expression of various antioxidant enzymes in corneal epithelial cells and found that GPx4 deficiency led to a significant increase in cytotoxicity compared to the silencing of other antioxidant enzymes. Although the remnant expression levels of each antioxidant enzymes after knockdown might be slightly different, the results might suggest the paramount importance of GPx4 as a defense mechanism in the corneal epithelium. In fact, even in the GPx4‐haplodeficient mice, a significant delay in epithelial wound repair was observed *in vivo*. In addition, these results were in contrast to those in our previous study, in which GPx4 and SOD1 were shown to be similarly important in conjunctival epithelial cells 24.

It is known that the byproducts of lipid hydroperoxide cause cell death and inhibition of cell proliferation 16, 17, and are considered to be implicated in pathologies of corneal diseases such as atopic keratoconjunctivitis and dry eye 8, 10. 4‐HNE is a major product generated during lipid peroxidation, and is a highly toxic molecule 16, 17. Recently, a distinctive iron‐dependent cell death, called ferroptosis has been primarily characterized in cancer cells and GPx4 is considered to be a central regulator of ferroptosis that is mediated by lipid peroxidation 32. In the present study, α‐tocopherol prevented lipid peroxidation and cell death due to GPx4 deficiency, and moreover, ferrostatin‐1 partially rescued decreased cell viability and increased LDH release by GPx4 knockdown. Our results suggest an implication of ferroptosis in the cytotoxicity and cell death in the GPx4‐deficient corneal epithelial cells. However, further investigations are necessary for the exact mechanism of cell death.

To the best of our knowledge, we first observed a delay in the corneal epithelial wound healing because of the lack of a specific antioxidant enzyme. It has been reported that dry eye phenotypes appear in aged SOD1 knockout mice 9. The researchers observed degeneration and dysfunction of lacrimal glands that have been speculated as causes of corneal epithelial damage 9. Although our *in vitro* data indicated that the loss of GPx4 in corneal epithelium led to impaired viability and delayed wound healing, an implication of dysfunctional lacrimal gland was not examined in GPx4^+/−^ mice. Another related report highlighted a delay in corneal epithelial wound healing in nuclear factor‐like 2 (Nrf2) mice 11. The Nrf2 protein is a transcription factor that regulates the expressions of numerous antioxidant enzymes and proteins. Therefore, the importance of the specific antioxidant enzyme was not the focus of the study, whereas the importance of Nrf2‐associated antioxidant defense mechanisms was clearly delineated.

In conclusion, our data demonstrated that GPx4 is a major antioxidant enzyme that is not only crucial for maintaining redox homeostasis but also for wound healing in corneal epithelial cells. Deficient GPx4 can aggravate the corneal pathology and may highlight a new therapeutic target for corneal disorders such as dry eye and keratoconjunctivitis. In addition, α‐tocopherol has a protective effect on lipid peroxidation, acting as an effective backup system for GPx4 in corneal epithelial cells.

## Author contributions

TU (Ueta) and OS conceived and designed the project and wrote the paper. OS and TU (Uchida) acquired the data. OS, TU (Ueta), and HI analyzed and interpreted the data.
